The article "Using a Selective Ensemble Support Vector Machine to Fuse Multimodal Features for Human Action Recognition" was published in 2022. Journal: Comput Intell Neurosci.

# Using a Selective Ensemble Support Vector Machine to Fuse Multimodal Features for Human Action Recognition

**DOI:** 10.1155/2022/1877464

**Published:** 2022-01-10

**Authors:** Chao Tang, Anyang Tong, Aihua Zheng, Hua Peng, Wei Li

**Affiliations:** ^1^School of Artificial Intelligence and Big Data, Hefei University, Hefei 230601, China; ^2^Anhui Provincial Key Laboratory of Multimodal Cognitive Computation, Anhui University, Hefei 230601, China; ^3^Department of Computer Science and Engineering, Shaoxing University, Shaoxing 312000, China; ^4^College of Information Science and Engineering, Jishou University, Jishou 416000, China; ^5^School of Computer and Information Engineering, Xiamen University of Technology, Xiamen 361024, China

## Abstract

The traditional human action recognition (HAR) method is based on RGB video. Recently, with the introduction of Microsoft Kinect and other consumer class depth cameras, HAR based on RGB-D (RGB-Depth) has drawn increasing attention from scholars and industry. Compared with the traditional method, the HAR based on RGB-D has high accuracy and strong robustness. In this paper, using a selective ensemble support vector machine to fuse multimodal features for human action recognition is proposed. The algorithm combines the improved HOG feature-based RGB modal data, the depth motion map-based local binary pattern features (DMM-LBP), and the hybrid joint features (HJF)-based joints modal data. Concomitantly, a frame-based selective ensemble support vector machine classification model (SESVM) is proposed, which effectively integrates the selective ensemble strategy with the selection of SVM base classifiers, thus increasing the differences between the base classifiers. The experimental results have demonstrated that the proposed method is simple, fast, and efficient on public datasets in comparison with other action recognition algorithms.

## 1. Introduction

Video has become the primary carrier of information owing to the rapid popularization and development of video acquisition equipment and broadband networks. With the massive emergence of video data, automating the procurement and analysis of the content has emerged as a problem that needs an urgent solution. The main purpose of HAR based on vision is to process and analyze the original image or image sequence data collected by the sensor (camera) via computer, to learn and understand the human action and behavior. HAR based on computer vision technology has been extensively used in several fields of human life, such as smart video surveillance [1, 2], human-machine interaction [3], robotics [3], video analytics [4], and human activity recognition [5–9].

Most of the existing human action recognition algorithms are based on the traditional RGB video data. However, human action recognition based on RGB information encounters multiple challenges as follows: (1) Complex background, occlusion, shadow, scale change, and different lighting conditions will induce tremendous difficulties for recognition, which is also the difficulty of action recognition based on RGB. (2) The same action will generate different views from different perspectives. (3) The same action performed by different people will be significantly varied, and two different types of action may have considerable similarity. These inherent defects of RGB visual information would limit the performance of human action recognition based on RGB information.

Recently, RGB-D cameras, such as Kinect v1 and v2 sensor by Microsoft, have made depth images available for human action recognition [5, 10, 11]. Each pixel in the depth image records the depth value of the scene, instead of light intensity. The introduction of depth camera expands the ability of the computer system to perceive the 3D visual world and makes up for the lack of dimensional information while 3D object information is captured as 2D visual information. Compared with RGB visual information, depth images can greatly reduce the influence of occlusion, complex background, and other factors by providing scene structure information. The color and texture are invariant under different illumination conditions. From a single perspective, if the different behaviors have similar 2D projections, the depth images can provide additional body shape information to distinguish different behaviors. Furthermore, Kinect also provides a powerful skeleton tracking algorithm, which can output the position of each 3D human joint point in real time. The skeleton joints of human body will not be affected by the changes of the scale and perspective.

According to the different types of input data, HAR technology based on RGB-D video can be roughly divided into three categories, namely, HAR based on RGB data, depth image data, and skeleton joints data.

### 1.1. Human Action Recognition Based on RGB Image Data

The early research on human action recognition based on RGB image sequence has been inspired by image processing technology, owing to the rich color and texture features of RGB image sequences. HAR is primarily carried out by extracting spatiotemporal interest points (STIP) in RGB video. Kovashka and Grauman [12] have proposed a human action recognition method based on hierarchical [13] model. This method combines HOG3D [14], HOG (histograms of oriented gradients), and HOF (histograms of optical flow) spatiotemporal domain descriptors and introduces a multicore learning model. Melfi et al. [15] have extended the Harris corner detection operator for video behavior recognition. First, the contour of the moving object is extracted, and then the 3D Harris points of interest are extracted from the moving object for HAR. In [16], the points of interest of the video frames are densely sampled in different scale spaces of the video frames to form dense trajectories. Thereafter, the features, namely, HOG, HOF, and MBH (motion boundary histogram), of the trajectories are extracted. Finally, SVM is used to classify the features.

Recently, owing to the development of machine learning theory, we can also use deep learning to extract features from RGB video data, besides utilizing the spatiotemporal interest points to extract the video image features.

Gammulle et al. [17] have obtained the video frame features through Convolutional Neural Networks (CNN) and then used the dual stream Long Short-Term Memory (LSTM) to train the features to realize HAR. Bilen et al. [18] have proposed to convert a video sequence into a dynamic image using the rank pool technology and further used CNN model to extract the features from the dynamic image for HAR. Arif et al. [19] have proposed the concept of motion graph. First, the 3D CNN network is used to extract video features, and thereafter the features of video frames are integrated into the motion map. Subsequent to these steps, the LSTM method is used to improve the accuracy of HAR. Majd and Safabakhsh [20] have first obtained the CNN features of the video frames through the CNN deep learning network. Thereafter, the CNN features are sent to the kernel cross correlation (KCC) filter to realize the automatic estimation of motion information.

Compared with the manually designed action features, although the video features are extracted automatically through deep learning, the accuracy of action recognition has increased. However, due to the unclear learning mechanism of deep learning, the stability of the extracted features is relatively poor, and a large number of parameter adjustment experiments need to be carried out manually. Therefore, the method based on deep learning has some limitations in practical application.

### 1.2. HAR Based on Depth Image

HAR based on depth image data primarily uses RGB image feature extraction method to extract the global and local features from the spatiotemporal volume. Compared with the RGB image, the depth image is not sensitive to illumination changes. Furthermore, it contains rich 3D structure information. However, the depth images also have some shortcomings. Owing to certain specific factors, such as specific materials, reflection, and interference, Kinect cannot estimate the depth of certain parts of the object in the scene. This results in the loss of part of the depth image obtained, forming several holes. Furthermore, the depth images obtained by Kinect lack the color features of objects, with abundant noises. These factors make it difficult to obtain robust features from depth images. Inspired by STIP feature extraction algorithm of RGB image sequence, Xia and Aggarwal [21] have obtained Depth Spatial Temporal Interest Points (DSTIP) of the depth image, by the two-dimensional Gaussian filtering and one-dimensional Gabor filtering. Based on this point of interest, the depth cuboid similarity features (DCSF) are extracted for HAR. Yang and Tian [22] have proposed a feature, namely, super normal vector, to represent the depth image sequence. The feature combines the local motion information and shape information in the depth image sequence and achieves outstanding experimental results on MSRDailyActivity3D and other datasets. Reza et al. [23] have proposed a weighted depth motion map (DMM) and then extracted the hog features from the weighted DMM for HAR.

Since the depth image lacks the description of the image color, texture, and other details, and the CNN neural network model is primarily intended to extract the color and texture features of the image, using CNN model to extract the features of depth image cannot achieve satisfactory results. Furthermore, the deep learning model needs a large amount of data for training. However, most of the depth image datasets have a small amount of data, which cannot be used for large-scale training using CNN and other neural networks. Hence the research output in this field is relatively small.

### 1.3. HAR Based on Skeleton Joints Data

The recognition of human action based on skeleton joint features can be traced back to the moving light display (MLD) experiment by Johansson et al. Owing to the limitation of sensors, the early description of the skeleton joint features results in the high noise of joint points, which leads to a low accuracy of HAR. Owing to the development of computer vision technology, particularly Kinect, people can get the robust joint points in real time. Yang and Tian [24] have proposed a bone feature representation method, which is obtained by the position difference of the skeleton nodes between different frames. First, three kinds of skeleton node position differences are extracted, which are the differences in static posture, motion, and offset. Thereafter, the three types of skeleton difference features are combined, and the EigenJoints features are obtained by the PCA dimension reduction. Finally, the action recognition is carried out by the naive Bayes classifier. Xia et al. [25] have proposed the usage of the histograms of 3D joints feature to realize the description of a skeleton action. The feature is to project the data of 12 main joints of the human body into the spherical coordinate system, then obtain their distribution histogram in the spherical coordinate system, and then use linear discriminant analysis to reduce the dimension of the obtained features. Finally, hidden Markov model is used to classify and express the features.

Researchers also try to use deep learning to learn features from human skeleton data. The main idea of this algorithm is to represent the human skeleton data into a suitable image form and then extract features from the skeleton image using CNN and other models for human action recognition. However, the constraints of the current deep learning theory make it very difficult to convert an appropriate skeleton image. Zhang et al. [26] have proposed Multilayer LSTM Networks for the skeleton feature learning and employed a smooth fractional fusion method to fuse the bone features of the multistream LSTM learning, which has improved the accuracy of the human action recognition. Li et al. [27] have proposed 3D skeleton-based action recognition using a novel symbiotic graph neural network, which handles action recognition and motion prediction jointly and uses graph-based operations to capture action patterns.

Briefly, despite the HAR methods based on state-of-the-art RGB-D having progressed tremendously, reliability of their applications in the realistic engineering scenarios is still modest. This is owing to the relatively large intraclass variations and small interclass differences of several actions, the variations in action speed, and the extreme computational complexities. This work fully utilizes the multimodal information acquired through a Kinect sensor to extract the features of human actions effectively. Moreover, an integrated multilearner strategy has been adopted for the classification to demonstrate exceptional generalizing capabilities.

The rest of this paper is organized as follows.  Section 2 presents a novel selective ensemble-based support vector machine (SESVM) approach to fuse the multimodal features for HAR.  Section 3 explains the extraction of multimodal features from RGB-D images by employing different methods. In Section 4, a selective ensemble-based SVM classification framework is deployed for feature recognition. The experimental results on the G3D dataset and Cornell Activity Dataset 60 are presented in Section 5, showing the feasibility and performance of the proposed approach. Finally, a brief conclusion and notes on further work are given in Section 6.

## 2. The Framework

The Kinect sensors produced by Microsoft can provide both RGB and depth information of the scene, in addition to the skeleton joint locations of human bodies. The depth images captured by Kinect sensor can provide light-invariant foreground information with depth geometry structure, and they have the advantages of texture, color invariance, and insensitivity to the influences from illumination, environment, and shadows. This paper utilizes multimodal data provided by the Kinect sensor and extracts three different features as the descriptors of the actions. Thus, an integrated multiclassifier algorithm is adopted for the classification to exploit the advantages of the different features.

Figure 1 shows the system configuration of the proposed approach. It achieves efficient computation from handling simple features while ensuring the robustness and recognition capability of the features. Particularly, our framework consists of the following steps:

1. Acquire synchronized RGB, depth, and joint images from the Kinect sensor
2. Convert the input RGB image to grayscale, and then extract the improved histogram of the oriented gradient features
3. Compute the depth motion map-based local binary pattern (DMM-LBP) from the depth image, and then extract joint-based hybrid joint features (HJFs) from the acquired 3D skeleton image
4. Train the selective ensemble-based support vector machine (SESVM) using the sample sets with combined features
5. Implement the same extraction process to the predicting images during action recognition, enter them into SESVM for recognition, and work out recognition result

The major contributions of this paper are summarized as follows:

1. A novel selective ensemble-based support vector machine (SESVM) method has been proposed to describe the human action features based on multimodal information. This method is capable of depicting human actions from the various points of view and has been verified by experiments on public datasets.
2. The improved RGB-based histogram of oriented gradient (RGB-HOG) features is adopted in this paper, which is invariant to geometric and optical deformations of the images.
3. The depth-based DMM-LBP features are created to maintain the dynamic characteristics of human actions with good local invariance.
4. The joint-based hybrid joint feature (HJF) has been adopted to provide the spatial structure information about human actions.
5. The correlation coefficient-based classifier selection algorithm (CCCSA) has been adopted to select classifiers from the existing ones for constructing the ensemble classifiers. This is for speeding up the prediction speed of the classifier, reducing the storage space requirements, and further improving the classification accuracy. By using fewer classifiers, the prediction speed can be accelerated because the computational overhead of prediction is reduced. In addition, due to the small number of individual classifiers in the selective ensemble learning system, the storage overhead is also reduced, because only a small number of individual models need to be saved.

## 3. Feature Extraction

This section introduces the feature extraction methods for various modalities. Particularly, Section 3.1 describes the improved HOG features for the RGB modality, Section 3.2 introduces the DMM-LBP features for the depth modality, and Section 3.3 explains the HJF features for the joint modality.

### 3.1. RGB-HOG Feature

Dalal and Triggs have first proposed the HOG feature to detect pedestrians in static images [28]. Thereafter, multiple researchers have presented the improved HOG features [29].

HOG algorithm is a feature extraction method recently used in the research of target recognition. However, the HOG feature extraction algorithm can only calculate the direction of information of a single gradient of pixels, which is not comprehensive enough, and has certain defects in describing the directional features of the target.

We have used the steerable filter algorithm which can obtain multidirectional information to make up for the deficiency of HOG algorithm. This method expands the single-directional information of a pixel to *N* multiple-directional information.

Freeman and Adelson [30] first proposed the steerable filter, which convolutes the image by generating templates in different directions to get the edge of the image. The convolution process increases the weight of the effective pixels and decreases the weight of invalid pixels by a weighting operation.

The general form of steerable filter is given as

(1) $$\begin{array}{c} G^{\alpha }=\sum_{i=1}^{N}k_{i}\left(\alpha \right)G_{i}, \end{array}$$

where *N* is the number of base filters and *G*_*i*_ the *i*th fundamental filter. Further, *k*_*i*_(*α*) represents the coefficients of the filter related to the direction degree *α*, and *G*^*α*^ is the filter in *α* direction.

We have used the method of obtaining multidirectional filter by the linear combination of a group of basic filters and the derivation of two-dimensional Gaussian function. The corresponding expression is given as

(2) $$\begin{array}{c} G\left(x,y\right)=k\left(\alpha \right)\exp\left[-\left(x^{2}+y^{2}\right)\right]. \end{array}$$

The specific expressions are given as

(3) $$\begin{array}{c} \left\{\begin{array}{c} G_{1}^{0}\left(x,y\right)=0.9213\left(2x^{2}-1\right)\exp\left[-\left(x^{2}+y^{2}\right)\right],\\ G_{1}^{\pi /3}\left(x,y\right)=1.843xy\;\exp\left[-\left(x^{2}+y^{2}\right)\right],\\ G_{1}^{2\pi /3}\left(x,y\right)=0.9213\left(2y^{2}-1\right)\exp\left[-\left(x^{2}+y^{2}\right)\right], \end{array}\right) \end{array}$$

and the corresponding coefficient is given as

(4) $$\begin{array}{c} \left\{\begin{array}{c} k_{1}\left(a\right)=\;\cos^{2}\;a,\\ k_{2}\left(a\right)=-2\;\cos\;a\;\sin\;a,\\ k_{3}\left(a\right)=\;\sin^{2}\;a, \end{array}\right) \end{array}$$

where *G*_1_^0^(*x*, *y*) and *G*_1_^2*π*/3^(*x*, *y*), respectively, represent the second derivative of image pixels in the corresponding direction, that is, the basis filter in the corresponding direction. The amplitude information in any direction can be calculated by the linear combination of the three expressions. The calculation formula after linear combination is shown as

(5) $$\begin{array}{c} G_{1}^{\alpha }=k_{1}\left(a\right)G_{1}^{0}\left(x,y\right)+k_{2}\left(a\right)G_{1}^{\pi /3}\left(x,y\right)+k_{3}\left(a\right)G_{1}^{2\pi /3}\left(x,y\right). \end{array}$$

We have combined the steerable filter algorithm with the traditional HOG algorithm. First, the steerable filter algorithm has been used to calculate the direction number and amplitude information with the highest direction value, and then the HOG algorithm is used to obtain the statistical direction histogram features. The algorithm flow, which shows the specific calculation, is depicted in Figure 2.

The implementation sequence of the HOG feature extraction algorithm can be described as follows:

*Step 1.* Normalize the Gamma space and the color space. To reduce the influence of illumination, the image needs to be normalized first. The contribution of local surface exposure to the texture strength is relatively large. Therefore, this type of compression can effectively reduce the local variations, in the shadow and illumination of the image. The image is first converted to grayscale as the color information contributes little. The Gamma compression formula is given as
  (6) $$\begin{array}{c} I\left(x,y\right)=I{\left(x,y\right)}^{\text{Gamma}}, \end{array}$$
where *I*(*x*, *y*) is the input RGB image. Gamma usually takes the value of 1/2.
*Step 2*. Let *p*(*x*, *y*) be the pixel of the gray image. Construct two mutually perpendicular directional controllable filters of *p* pixel (the directions of the filters are *α* and *β*, respectively, and *α*+*β*=*π*/2), and record them as *F*^(*α*)^ and *F*^(*β*)^, respectively. Then, the gradient values of point *p* in *α* and *β* directions are given as
  (7) $$\begin{array}{c} \left\{\begin{array}{c} G_{\alpha }\left(x,y\right)=F^{\left(\alpha \right)}*I\left(x,y\right),\\ G_{\beta }\left(x,y\right)=F^{\left(\beta \right)}*I\left(x,y\right). \end{array}\right) \end{array}$$
*Step 3*. Compute the gradient of the image. Compute the gradient in the directions of the horizontal and vertical axes that are the gradient orientation of each pixel. The computation of derivatives can capture the contours, human figures, and certain texture information from the image, besides further reducing the influence from illumination. The gradient of a pixel (*x*, *y*) in the image is given as
  (8) $$\begin{array}{c} \left|\nabla G\left(x,y\right)\right|=\sqrt{G_{\alpha }{\left(x,y\right)}^{2}+G_{\beta }{\left(x,y\right)}^{2}},\\ \theta \left(x,y\right)=\tan^{-1}\left(\frac{G_{\beta }\left(x,y\right)}{G_{\alpha }\left(x,y\right)}\right), \end{array}$$
where *G*_*x*_(*x*, *y*), *G*_*y*_(*x*, *y*), *G*(*x*, *y*), and *θ*(*x*, *y*) are the horizontal gradient, the vertical gradient, the gradient amplitude, and the gradient angle at pixel (*x*, *y*), respectively.
*Step 4*. Construct a histogram of the oriented gradient for each cell. This provides coding for the local image area and is capable of maintaining the invariance to human postures and appearances in the image. We divide the image into a number of “unit cells,” and each cell contains 6 *∗* 6 pixels, for instance. Suppose that we use a 9-bin histogram to collect the gradient information of these 6 *∗* 6 pixels, i.e., to divide the gradient orientation of the cell of 360 degrees into nine oriented blocks. For example, if the gradient orientation of the pixel is 20–40 degrees, then the 2nd histogram bin count will be increased by 1. By doing so, every pixel in the cell is projected with a weight onto the histogram by its gradient orientation (mapped into specific angle range). Consequently, the histogram of the oriented gradient of the cell is obtained, which is the 9D feature vector of the cell (since there are nine bins).
*Step 5*. Concatenate cells into blocks and normalize the oriented gradient histograms within each block. The strength of the gradient changes significantly owing to the variations in the local illumination strength and foreground and background contrast. Hence, the gradient strength needs to be normalized. The normalization can further compress the illumination, shadow, and edges. The implementation sequence is as follows: (1) to combine the unit cells into large and spatially connected blocks; (2) to concatenate feather vectors from all cells in the block to generate the HOG feature of the block. Since there are overlapping among the blocks, feature vector of each cell may appear in the final feature vector multiple times. We call this normalized block descriptor (vector) “the HOG descriptor.”
*Step 6*. Collect the HOG features. This last step is to collect the HOG features from all overlapping blocks in the testing window and combine them into the final feature vector to be used in the classification.

(9) $$\begin{array}{c} x^{\text{RGB}-\text{HOG}}=\left[x_{1},x_{2},\ldots ,x_{m}\right]. \end{array}$$

### 3.2. DMM-LBP Feature

With the development of RGB-D camera, several action recognition algorithms based on the depth image have been proposed. Depth image can be used to represent the 3D structure and shape information of objects. The depth image is projected onto three orthogonal planes [31] to form a depth motion map, and then the gradient histogram is extracted as the action feature. Specifically, using the front view, top view, and left view, the human body is positioned in the Cartesian coordinate system. Further, the depth data of the human body is projected to the front view, top view, and left view, respectively. Each frame action can be expressed as *V*={front, top, left}, where front, top, and left represent the human projection in the front view, top view, and left view, respectively. For the depth data video of *N* frames, the DMM features are calculated as

(10) $$\begin{array}{c} {\text{DMM}}_{V}=\sum_{i=s}^{e}\left|{\text{MAP}}_{V}^{i}-{\text{MAP}}_{V}^{i-1}\right|, \end{array}$$

where *i* is the time sequence frame. MAP_*V*_^*i*^ represents the projection of frame *i* on view *V*, and *s* and *e* represent the start frame and the end frame, respectively.

Several pixel values in the depth image are 0, which is not helpful for the description of action features. Hence, the region of interest operation should be performed for each frame image. To further filter the pixels in DMM, the local binary pattern (LBP) operation is performed on DMM. LBP is an effective texture feature description operator. It was first proposed by Ojala et al. [32]. It is used to extract texture features. Its advantage is that it has high robustness to the changes of illumination and rotation, and the extracted features are the local texture features of the image.

For a given point DMM_*V*_(*x*_*c*_, *y*_*c*_) on the image DMM_*V*_(*x*, *y*), LBP can be calculated as

(11) $$\begin{array}{c} {\text{DMM}}_{V}-\text{LBP}\left(x_{c},y_{c}\right)=\sum_{i=1}^{m}T\left({\text{DMM}}_{V}\left(x_{i},y_{i}\right)-{\text{DMM}}_{V}\left(x_{c},y_{c}\right)\right)2^{i},\\ T\left(x\right)=\left\{\begin{array}{c} 1,\;x\geq 0,\\ 0,\;x\leq 0, \end{array}\right) \end{array}$$

where *m* is number of sampling points. The coordinates of *f*(*x*_*i*_, *y*_*i*_)_*i*=1_^*m*^ can be expressed as

(12) $$\begin{array}{c} \left(x_{c}-r\;\sin\left(\frac{2\pi i}{m}\right),y_{c}+r\;\cos\left(\frac{2\pi i}{m}\right)\right), \end{array}$$

where *r* is the sampling radius of pixel *f*(*x*_*c*_, *y*_*c*_).

The LBP feature extraction algorithm of depth image is as follows:

*Step 1*. The region of interest of the depth image is extracted as the detection window.
  (13) $$\begin{array}{c} d\left(x,y\right)\leftarrow \text{ROI}\left(D\left(x,y\right)\right). \end{array}$$
*Step 2*. Get the projection view of the depth map in three different directions.
  (14) $$\begin{array}{c} {\text{MAP}}_{V}\left\{V=\text{front},\text{top},\text{left}\right\}\leftarrow d\left(x,y\right). \end{array}$$
*Step 3*. The depth motion map is calculated from the projection view.
  (15) $$\begin{array}{c} {\text{DMM}}_{V}=\sum_{i=s}^{e}\left|{\text{MAP}}_{V}^{i}-{\text{MAP}}_{V}^{i-1}\right|. \end{array}$$
*Step 4*. Divide the detection window into 16*∗*16 cells.
  (16) $$\begin{array}{c} {\text{Cell}}_{i}\left(x,y\right)\left(i=1,2,\ldots ,16\right)\leftarrow {\text{DMM}}_{V}\left(x,y\right). \end{array}$$
*Step 5*. For a pixel in each Cell_*i*_(*x*, *y*), the pixel value of its adjacent eight pixels is compared with it. If the value of the surrounding pixels is greater than the value of the center pixel, the position of the pixel is marked as 1; otherwise, it is 0. Accordingly, the eight points in the 3*∗*3 domain can be compared to generate 8 bit binary number; that is, the LBP value of the center pixel of the window can be obtained.
  (17) $$\begin{array}{c} {\text{LBP}}_{i}\left(x,y\right)\leftarrow {\text{Cell}}_{i}\left(x,y\right)\left(i=1,2,\ldots ,16\right). \end{array}$$
*Step 6*. Calculate the histogram of each cell, i.e., the frequency of each number, and normalize the histogram.
  (18) $$\begin{array}{c} {\text{LBPhog}}_{i}\leftarrow \text{BinCount}\left({\text{LBP}}_{i}\left(x,y\right),\;i=1,2,\ldots ,16\right). \end{array}$$
*Step 7*. Finally, the statistical histogram of each cell is connected into a feature vector, which is the LBP feature vector of the whole depth image.

(19) $$\begin{array}{c} x^{\text{DMM}-\text{LBP}}\leftarrow \left\{{\text{LBPhog}}_{1},{\text{LBPhog}}_{2},\ldots ,{\text{LBPhog}}_{16}\right\}\\ x^{\text{DMM}-\text{LBP}}=\left[x_{1},x_{2},\ldots ,x_{n}\right]. \end{array}$$

DMM-LBP feature extraction algorithm flow is shown in Figure 3.

### 3.3. HJF Feature

RGB-D sensor can quickly obtain the human joint position and three-dimensional skeleton through the depth image information. These data contain rich information, which brings new ideas and methods to HAR. For example, Microsoft released Kinect v2 that provides us with the information of 20 human 3D bone points and then extracts the features of these information points. Further, the feature dimension will become minuscule, which is conducive to speeding up the calculation and improving the real time performance.

Different human actions are reflected not only in the difference of joint position information but also in the energy features of the joint point sequence. We have used the joint kinetic energy features, direction change features, and joint potential energy features as the hybrid joint features.

To calculate the kinetic energy information of the human joint points, it is necessary to obtain the three-dimensional coordinates of the human joint points *P*(*x*, *y*, *z*). Therefore, according to the coordinate information changes of the two adjacent frames, the kinetic energy of the human joint points in each frame is calculated as

(20) $$\begin{array}{c} {\text{KEF}}_{i,t}=\frac{1}{\Delta s^{2}}k\left|P_{i,t}\left(x_{i,t},y_{i,t},z_{i,t}\right)-P_{i,t-\Delta t}\left(x_{i,t-\Delta t},y_{i,t-\Delta t},z_{i,t-\Delta t}\right)\right|\\ =\frac{1}{\Delta s^{2}}k\left\{{\left(x_{i,t}-x_{i,t-\Delta t}\right)}^{2}+{\left(y_{i,t}-y_{i,t-\Delta t}\right)}^{2}+{\left(z_{i,t}-z_{i,t-\Delta t}\right)}^{2}\right\}, \end{array}$$

where KEF_*i*,*t*_ is the kinetic energy of the *i*th joint in *F*_*t*_ frame and *k* is the kinetic energy parameter. In the experiment, *k* can be taken as 1. Δ*t* is the time interval between the two adjacent frames.

Human action is related to the information of the current and past positions. In different action states, the speed of movement of the joints randomly varies with time, and the direction of change may also vary. According to the coordinates of human 3D joint points, the direction change vector of each joint point is calculated as the human motion feature, given as

(21) $$\begin{array}{c} {\text{DC}}_{i,t}=\left(x_{i,t}-x_{i,t-1},y_{i,t}-y_{i,t-1},z_{i,t}-z_{i,t-1}\right), \end{array}$$

where DC_*i*,*t*_ represents the direction change vector of the *i*th joint point in the *F*_*t*_ frame relative to the *i*th joint point in the previous *F*_*t*−1_ frame. Further, *x*_*i*,*t*_, *y*_*i*,*t*_, and *z*_*i*,*t*_ represent the spatial three-dimensional coordinates of the joint point in the *F*_*t*_ frame.

We have combined the features of the joint kinetic energy and joint direction change into a new feature, which is defined as the hybrid joint feature, given below

(22) $$\begin{array}{c} x^{\text{HJF}}\leftarrow \left\{{\text{KEF}}_{1},{\text{KEF}}_{2},\ldots ,{\text{KEF}}_{20},{\text{DC}}_{1},{\text{DC}}_{2},\ldots ,{\text{DC}}_{20}\right\},\\ x^{\text{HJF}}=\left[x_{1},x_{2},\ldots ,x_{q}\right]. \end{array}$$

### 3.4. Feature Fusion

Feature fusion is an effective method to clearly distinguish human action features. Currently, the major feature fusion methods include the pixel-level, feature-level, and decision-level fusions. We employ the feature-level fusion in this study, which is able to retain and fuse the effective recognizable information of the features, besides effectively eliminating the redundant feature information and features with poor distinctiveness. Particularly, RGB-HOG, DMM-LBP, and HJF features are fused into the descriptive features of action, i.e.,

(23) $$\begin{array}{c} \text{RDH}=\left(\text{RGB}-\text{HOG},\text{DMM}-\text{LBP},\text{HJF}\right). \end{array}$$

Compared with the single action features, these composite features show excellent robustness as they are a collection of the advantages of every single feature and more suitable for describing the human action features.

## 4. Recognition Method

Recently, the research on the theory and algorithm of the ensemble learning has been a hotspot in the field of machine learning. The construction of an ensemble learning machine is divided into two steps, namely, the generation step and the merging step. The key is to effectively generate a base learning machine with strong generalization ability and great differences. Alternatively, the accuracy and diversity of the base learning machines are two important factors. In general, the predictive effect of the ensemble learning machine is significantly better than that of the single base learning machine. However, the predictive speed of the ensemble learning machine is significantly slower than that of the single base learning machine. Moreover, as the number of the base learning machines increases, the needed storage space increases sharply, which is a serious problem for online learning. Zhou et al. [33] have proposed the “selective ensemble” to eliminate the basic learners with poor performance and, hence, to select certain ones to build the set for better prediction effect.

We propose a selective ensemble-based SVM classification framework for recognition. Assuming that *T*_*Tr*_={(**x**_*i*_, *y*_*i*_)}_*i*=1_^*N*_*Tr*_^ is a given training set for each training sample (*x*_*i*_, *y*_*i*_), its input variable is action feature vector **x**_*i*_=(*x*_*i*1_, *x*_*i*2_,…, *x*_*iM*_) ∈ *R*^*M*^, output variable is action category *y*_*i*_ ∈ Ω={*ω*_1_, *ω*_2_,…, *ω*_*c*_}, and *c* is the number of action classes. At the same time, let *T*_Val_={(**x**_*i*_, *y*_*i*_)}_*i*=1_^*N*_Val_^ denote verification set with the capacity of *N*_Val_.  Table 1 shows the selective ensemble-based SVM classification algorithm (SESVM).

Selective ensemble learning assumes that the multiple base learning machines have been generated, and only some of them are selected to construct the final ensemble based on a certain selection strategy. In the selective ensemble learning, diversity among the base classifiers plays an important role in explaining the working mechanism of multiclassifier systems and constructing effective ensemble systems. Current diversity measures can be divided into two kinds, namely, (i) the paired diversity measures for calculating the diversity between two basic classifiers and (ii) the unpaired diversity measures targeted at all basic classifiers. Paired diversity measures include *Q* statistics, correlation coefficient, disagreement measure, and double error measure. Disagreement measure method is used in this study as it features simple calculation, wide application, and favorable results in most cases. Suppose that SVM_*i*_ and SVM_*j*_ are two different classifiers whose relationship is given in Table 2.

The measurement of correlation coefficient *ρ*_*i*,*j*_ can be defined as

(24) $$\begin{array}{c} \rho_{i,j}\left({\text{SVM}}_{i},{\text{SVM}}_{j}\right)=\frac{N^{11}N^{00}-N^{10}N^{01}}{\sqrt{\left(N^{11}+N^{10}\right)\left(N^{01}+N^{00}\right)\left(N^{11}+N^{01}\right)\left(N^{10}+N^{00}\right)}}. \end{array}$$

Table 3 shows the correlation coefficient-based classifier selection algorithm (CCCSA). Accordingly, when there are two or more values that are equal and minimal in {Err^(1)^, Err^(2)^, Err^(3)^, Err^(4)^}, there should be a priority ranking in {*A*^(0)^, *A*^(1)^, *A*^(2)^, *A*^(3)^}, which is *A*^(3)^ > *A*^(2)^ > *A*^(1)^ > *A*^(0)^, e.g., *A* ← *A*^(3)^ when Err^(3)^ and Err^(2)^ are equal. After obtaining the filtered base classifier set, the key problem is the output of the combined decision-making. In terms of the fusion decision output of the multiple classifier systems, there are two methods [34], namely, class label-based decision output method and support function fusion-based decision output method.

We have adopted the majority voting based on the confidence owing to the simplicity and effectiveness of the class label fusion. Each classifier has been considered as totally equal in the simple voting method, which however may differ in practice. Thus, the classifiers with poorer performance have been given smaller weights while those with better performance have been given larger weights in majority voting based on confidence. Base classifiers set *A*={SVM_1_^*∗*^, SVM_2_^*∗*^,…, SVM_*N*_^*∗*^} have been obtained after being screened by CCCSA. Then, the voting weight of each basic classifier has been determined based on its precision. The voting weight of a basic classifier SVM_1_^*∗*^ depends on its error rate*ε*_*i*_, which is defined as

(25) $$\begin{array}{c} \varepsilon_{i}=\frac{1}{N}\sum_{i=1}^{N}I\left({\text{SVM}}_{i}^{*}\left(x_{i}\right)\neq y_{i}\right). \end{array}$$

Note that if the predicate *p* : SVM_*i*_^*∗*^(**x**_*i*_) ≠ *y*_*i*_ is true, *I*(*p*)=1; otherwise, it is 0. The weight of the basic classifier SVM_*i*_^*∗*^ can be defined as

(26) $$\begin{array}{c} w_{i}=\frac{1}{2}\ln\left(\frac{1-\varepsilon_{i}}{\varepsilon_{i}}\right). \end{array}$$

If *ε*_*i*_ approaches 0, then *w*_*i*_ is a large value. If *ε*_*i*_ approaches 1, then *w*_*i*_ is a large negative value. The classification result of the set of *N* classifiers SVM^*∗*^(**x**) is given as

(27) $$\begin{array}{c} \underset{y}{\text{Result}\leftarrow \arg\max}\frac{1}{N}\sum_{i=1}^{N}w_{i}*{\text{SVM}}_{i}\left(x\right). \end{array}$$

## 5. Experimental Results

In this section, the experiments are conducted using the G3D dataset and Cornell Activity Dataset 60. Both the results and analyses have been presented to show the feasibility and performance of the proposed approach.

### 5.1. Datasets

G3D dataset [35] contains 20 categories of human actions, each of which has been performed by 10 persons. The 20 category actions are punch right, punch left, kick right, kick left, defend, golf swing, tennis swing forehand, tennis swing backhand, tennis serve, throw bowling ball, aim and fire gun, walk, run, jump, climb, crouch, steer a car, wave, flap, and clap. Cornell Activity Dataset 60 (CAD60) [36] contains 12 actions, which are performed by 4 persons in 5 different environments. These actions are rinsing mouth, brushing teeth, wearing contact lens, talking on phone, drinking water, opening container, chopping, stirring, talking on couch, relaxing on couch, writing on whiteboard, and working on computer. The action in G3D dataset and CAD60 contains image information in three different models, namely, RGB image, depth image, and skeleton joint image, as illustrated in Figures 4 and 5.

### 5.2. Experiments and Results

In this section, we validate the feasibility and efficiency of the proposed method in two experiments. Cross-validation has been adopted in the experiments to train the classification model and to test its performance. First, we test the recognition rate on the G3D dataset and CAD60, based on the single feature and the algorithm in this paper. In the second experiment, we compare our method to alternative algorithms. The result of the first experiment is presented using the confusion matrix. The element (*i*, *j*) is the percentage of actions of class *i* that are classified as actions of class *j*. Therefore, the classification result is better for larger numbers of diagonal elements.

In Figures 6–8, the recognition rates using the single feature on the G3D dataset have been illustrated with a confusion matrix.  Figure 9 is the recognition rate of the proposed method using multimodal fusion information. From the experimental results shown in Figures 6–9, we can see that the recognition accuracy using combined features is higher than that using single features. This shows that the representation of human action feature directly affects the recognition effect of human action recognition methods. Single feature is often affected by human appearance, environment, camera setting, and other factors, and the recognition effect is limited. From Figure 9, we can see that the recognition rate of four actions (defend, tennis serve, throw bowing ball, and clap) is 100%, and the recognition rate of three actions (walk, run, and jump) is low and easy to confuse. Through the analysis, it is found that for actions such as walk, run, and jump, the action feature that can really distinguish these actions is the motion frequency, which needs to use the correlation between the information of multiple frames and the characteristics of adjacent frames when training the action model.

In Figures 10–12, the recognition rate using the single modal feature on the CAD60 has been illustrated with the confusion matrix.  Figure 13 shows the recognition rate of the proposed method using multimodal features on the CAD60. Through comparison, it is obvious that the proposed method achieves a good recognition rate of 91.7% on CAD60.

Table 4 shows the recognition rates using the single modal feature and multimodal features in terms of precision. It can be observed that the recognition rates of the proposed method using multimodal features are higher than the recognition rates of those methods using the single modal feature.

In the second experiment, we have compared the proposed method to alternative ones.  Table 5 shows the comparison between our algorithm, boosting, bagging, support vector machine (SVM), and artificial neural networks (ANNs). Accordingly, the integrated multilearner recognition algorithm based on multimodal features has achieved the highest recognition rate of 92%.

Table 6 compares the average class accuracy of our method with results reported by other researchers. Compared with the existing approaches, our method outperforms the state-of-the-art approaches. Note that a precise comparison between the approaches is difficult, since experimental set-ups, e.g., different strategy in training, slightly differ with each approach.

## 6. Conclusion

This paper presents a novel approach to HAR, which is a challenging research topic. A Kinect sensor has been deployed to acquire RGB-D image data, and the multimodal features (RGB-HOG features, DMM-LBP features, and HJF features) were extracted. The selective ensemble-based support vector machine (SESVM) has been adopted to fully utilize the biasing effects from different learners. The experiments have been conducted on standard public datasets and achieved good recognition rates. However, a large number of tagged video training samples is required for the classifier to achieve a good generalizing capability. This demands abundant manual tagging work and thus increases the practical difficulties. Therefore, our future work will focus on the utilization of the abundant untagged video samples in hand, to enhance the system performance.

## Figures and Tables

**Figure 1:** The proposed system configuration.

**Figure 2:** The algorithm flow of HOG algorithm.

**Figure 3:** DMM-LBP feature extraction algorithm flow.

**Figure 4:** Sample images from the G3D dataset. (a) RGB image. (b) Depth image. (c) Skeleton joint image.

**Figure 5:** Sample images from the Cornell Activity Dataset 60. (a) Depth image. (b) RGB image. (c) Skeleton joint image.

**Figure 6:** The confusion matrix based on RGB-HOG features on the G3D dataset.

**Figure 7:** The confusion matrix based on DMM-LBP features on the G3D dataset.

**Figure 8:** The confusion matrix based on HJF on the G3D dataset.

**Figure 9:** The confusion matrix based on this paper's method on the G3D dataset.

**Figure 10:** The confusion matrix based on RGB-HOG features on the CAD60.

**Figure 11:** The confusion matrix based on DMM-LBP features on the CAD60.

**Figure 12:** The confusion matrix based on HJF on the CAD60.

**Figure 13:** The confusion matrix based on the method of this paper on the CAD60.

**Table 1:** SESVM.

**Input**:
Training set *T*_*Tr*_={(**x**_*i*_, *y*_*i*_)}_*i*=1_^*N*_*Tr*_^, verification set *T*_Val_={(**x**_*i*_, *y*_*i*_)}_*i*=1_^*N*_*Val*_^, base classification algorithm SVM, number of base classifiers *M*, number of selected base classifiers *N*
**Output**:
Selected base classifier set {SVM_1_^*∗*^, SVM_2_^*∗*^,…, SVM_*N*_^*∗*^}
**Training process**:
(1) Initialize the base classifier set Θ=∅
(2) **For***m*=1,2,…, *M*
(3) Based on the training set *T*_*Tr*_={(**x**_*i*_, *y*_*i*_)}_*i*=1_^*N*_*Tr*_^, a new training set *T*_*Tr*_^(*m*)^ is obtained by using Bootstrap random sampling method
(4) The base classifier SVM_*m*_ is trained on the training set *T*_*Tr*_^(*m*)^ by using the base classification algorithm SVM and added to the set Θ
(5) **End for**
(6) Selecting process:
(7) Each base classifier SVM_*m*_(*m*=1,2,…, *M*) is tested on verification set *T*_Val_={(**x**_*i*_, *y*_*i*_)}_*i*=1_^*N*_Val_^ and its output *O*_*m*_(*m*=1,2,…, *M*) is obtained
(8) The selected base classifier set is obtained by using CCCSA
{SVM_1_^*∗*^, SVM_2_^*∗*^,…, SVM_*N*_^*∗*^} ← CCCSA(SVM_*m*_(*m*=1,2,…, *M*))

**Table 2:** Classifiers' relational table of classification of the samples.

Relations	SVM_*i*_ correct classification (1)	SVM_*i*_ incorrect classification (0)
SVM_*j*_ correct classification (1)	*N* ^11^	*N* ^10^
SVM_*j*_ incorrect classification (0)	*N* ^01^	*N* ^00^

*Note*. *N*^*AB*^ is the number of samples in the dataset, classified correctly (*A* = 1) or incorrectly (*A* = 0) by SVM_*i*_, and correctly (*B* = 1) or incorrectly (*B* = 0) by SVM_*j*_.

**Table 3:** CCCSA.

**Input**: The basic classifier set *A*={SVM_1_, SVM_2_,…, SVM_*M*_}, the diversity threshold *λ*, the verification set *T*_Val_={(**x**_*i*_, *y*_*i*_)}_*i*=1_^*N*_Val_^, the number of base classifiers set crad(*A*) and selective ensemble scale *N*
**Process**:
(1) **While** (crad(*A*) > *N*&&∀*ρ*_*i*,*j*_(SVM_*i*_, SVM_*j*_)(*i* ≠ *j*) {
(2)*A*^(0)^ ← *A*
(3)*A*^(1)^ ← {*A|*SVM_*i*_ ∉ *A*}
(4)*A*^(2)^ ← {*A|*SVM_*j*_ ∉ *A*}
(5)*A*^(3)^ ← {*A|*SVM_*i*_, SVM_*j*_ ∉ *A*}
(6) The error rates of *A*^(0)^, *A*^(1)^, *A*^(2)^, and*A*^(3)^ on verification set *T*_Val_ were calculated, with the min error rates saved
Err^(0)^ ← ERR(*A*^(0)^, *T*_Val_), Err^(1)^ ← ERR(*A*^(1)^, *T*_Val_),
Err^(2)^ ← ERR(*A*^(2)^, *T*_Val_), Err^(3)^ ← ERR(*A*^(3)^, *T*_Val_)
(7)Min − err ← MIN(Err^(0)^, Err^(1)^, Err^(2)^, Err^(3)^)
(8) **if**(Min − err*==*Err^(0)^)*A* ← *A*^(0)^
(9) **else if**(Min − err*==*Err^(1)^)*A* ← *A*^(1)^
(10) **else if**(Min − err*==*Err^(2)^)*A* ← *A*^(2)^
(11) **Else***A* ← *A*^(3)^
(12) **end**}
(13)*A*^*∗*^ ← *A*;
**Output**: The selected base classifier set *A*^*∗*^

**Table 4:** Recognition rate using the single modal feature and multimodal features.

Dataset	Descriptor	Precision (%)
G3D	RGB-HOG	83.7
	DMM-LBP	83.2
	HJF	83.7
	Mixed features	91.7

CAD60	RGB-HOG	85.3
	DMM-LBP	86.0
	HJF	88.6
	Mixed features	91.8

**Table 5:** The comparison results between the proposed method and other machine learning methods.

Dataset	Descriptor	SESVM (%)	Boosting (%)	Bagging (%)	SVM (%)	ANNs (%)
G3D	RGB-HOG	83.7	83.2	75.2	80.2	74.2
	DMM-LBP	83.2	82.4	79.4	83.4	80.2
	HJF	83.7	84.0	80.5	83.6	74.4
	Mixed features	91.7	89.5	83.2	87.7	82.4

CAD60	RGB-HOG	85.3	87.3	80.0	82.0	76.2
	DMM-LBP	86.0	87.4	79.2	84.3	80.5
	HJF	88.6	89.2	80.2	84.4	74.2
	Mixed features	91.8	89.1	83.3	87.6	82.2

**Table 6:** The comparison results between our approach and other methods.

Researchers	Descriptor	Recognition methods	Accuracy	
			G3D (%)	CAD60 (%)
Dollár et al. [37]	Sparse	SVM	78	83
	Spatiotemporal features			
Liu et al. [38]	PMI spatiotemporal features	SVM	82	86
Laptev et al. [39]	Spatiotemporal corner	SVM	87	84
Rapantzikos et al. [40]	Dense saliency spatiotemporal features	KNN	88	89
Rodriguez et al. [41]	Spatiotemporal template	Template matching	88	89
Our approach	Mixed features	SESVM	91.7	91.8

## Data Availability

The data used to support the findings of this study are available from the corresponding author upon request.

## References

[1] Tosato D., Spera M., Cristani M., Murino V. (2013). Characterizing humans on riemannian manifolds. *IEEE Transactions on Pattern Analysis and Machine Intelligence*.

[2] Ladjailia A., Bouchrika I., Harrati N., Mahfouf Z. (2018). *Encoding Human Motion for Automated Activity Recognition in Surveillance Applications*.

[3] Theodoridis T., Agapitos A., Hu H., Lucas S. M. (2008). Ubiquitous robotics in physical human action recognition: a comparison between dynamic ANNs and GP. *IEEE International Conference on Robotics and Automation*.

[4] Chen C., Liu K., Jafari R., Kehtarnavaz N. Home-based senior fitness test measurement system using collaborative inertial and depth sensors.

[5] Chen C., Jafari R., Kehtarnavaz N. (2017). A survey of depth and inertial sensor fusion for human action recognition. *Multimedia Tools and Applications*.

[6] Das Dawn D., Shaikh S. H. (2016). A comprehensive survey of human action recognition with spatio-temporal interest point (STIP) detector. *The Visual Computer*.

[7] Lim C. H., Vats E., Chan C. S. (2015). Fuzzy human motion analysis: a review. *Pattern Recognition*.

[8] Lo Presti L., La Cascia M. (2016). 3D skeleton-based human action classification: a survey. *Pattern Recognition*.

[9] Ziaeefard M., Bergevin R. (2015). Semantic human activity recognition: a literature review. *Pattern Recognition*.

[10] Cai Z., Han J., Liu L., Shao L. (2017). RGB-D datasets using microsoft kinect or similar sensors: a survey. *Multimedia Tools and Applications*.

[11] Zhang J., Li W., Ogunbona P. O., Wang P., Tang C. (2016). RGB-D-based action recognition datasets: a survey. *Pattern Recognition*.

[12] Kovashka A., Grauman K. Learning a hierarchy of discriminative space-time neighborhood features for human action recognition.

[13] Attique Khan M., Alhaisoni M., Armghan A. (2021). Video analytics framework for human action recognition. *Computers, Materials and Continua*.

[14] Klser A., Marszalek M., Schmid C. A spatio-temporal descriptor based on 3D-gradients.

[15] Melfi R., Kondra S., Petrosino A. (2013). Human activity modeling by spatio temporal textural appearance. *Pattern Recognition Letters*.

[16] Wang H., Kläser A., Schmid C., Liu C.-L. (2013). Dense trajectories and motion boundary descriptors for action recognition. *International Journal of Computer Vision*.

[17] Gammulle H., Denman S., Sridharan S., Fookes C. Two stream LSTM: a deep fusion framework for human action recognition.

[18] Bilen H., Fernando B., Gavves E., Vedaldi A. (2018). Action recognition with dynamic image networks. *IEEE Transactions on Pattern Analysis and Machine Intelligence*.

[19] Arif S., Wang J., Ul Hassan T., Fei Z. (2019). 3D-CNN-based fused feature maps with LSTM applied to action recognition. *Future Internet*.

[20] Majd M., Safabakhsh R. (2019). A motion-aware ConvLSTM network for action recognition. *Applied Intelligence*.

[21] Xia L., Aggarwal J. K. Spatio-temporal depth cuboid similarity feature for activity recognition using depth camera.

[22] Yang X., Tian Y. Super normal vector for activity recognition using depth sequences.

[23] Reza A., Maryam A. A., Shohreh K., Sergio E. (2019). Dynamic 3D hand gesture recognition by learning weighted depth motion maps. *IEEE Transactions on Circuits and Systems for Video Technology*.

[24] Yang X., Tian Y. L. EigenJoints-based action recognition using Nave-Bayes-Nearest-Neighbor.

[25] Xia L., Chen C. C., Aggarwal J. K. View invariant human action recognition using histograms of 3D joints.

[26] Zhang S., Yang Y., Xiao J. (2018). Fusing geometric features for skeleton-based action recognition using multilayer LSTM networks. *IEEE Transactions on Multimedia*.

[27] Li M., Chen S., Chen X., Zhang Y., Wang Y., Tian Q. (2021). Symbiotic graph neural networks for 3D skeleton-based human action recognition and motion prediction. *IEEE Transactions on Pattern Analysis and Machine Intelligence*.

[28] Dalal N., Triggs B. Histograms of oriented gradients for human detection.

[29] Chowdhury S. A., Uddin M. N., Kowsar M. M. S., Deb K. Occlusion handling and human detection based on histogram of oriented gradients for automatic video surveillance.

[30] Freeman W. T., Adelson E. H. (1991). The design and use of steerable filters. *IEEE Transactions on Pattern Analysis and Machine Intelligence*.

[31] Yang X., Zhang C., Tian Y. L. Recognizing actions using depth motion maps-based histograms of oriented gradients.

[32] Ojala T., Pietikainen M., Harwood D. Performance evaluation of texture measures with classification based on Kullback discrimination of distributions.

[33] Zhou Z.-H., Wu J., Tang W. (2002). Ensembling neural networks: many could be better than all. *Artificial Intelligence*.

[34] Wozniak M., Grana M., Corchado E. (2014). A survey of multiple classifier systems as hybrid systems. *Information Fusion*.

[35] Bloom V., Argyriou V., Makris D. (2016). Hierarchical transfer learning for online recognition of compound actions. *Computer Vision and Image Understanding*.

[36] Oreifej O., Liu Z. Hon4d: histogram of oriented 4d normals for activity recognition from depth sequences.

[37] Dollár P., Rabaud V., Cottrell G., Belongie S. Behavior recognition via sparse spatio-temporal features.

[38] Liu J., Luo J., Shah M. Recognizing realistic actions from videos “in the wild”.

[39] Laptev I., Marszalek M., Schmid C., Rozenfeld B. Learning realistic human actions from movies.

[40] Rapantzikos K., Avrithis Y., Kollias S. Dense saliency-based spatiotemporal feature points for action recognition.

[41] Rodriguez M. D., Ahmed J., Shah M. Action MACH a spatio-temporal maximum average correlation height filter for action recognition.

